This article has been retracted.

# Improvement of Landfill Leachate Biodegradability with Ultrasonic Process

**DOI:** 10.1371/journal.pone.0027571

**Published:** 2012-07-19

**Authors:** Amir Hossein Mahvi, Ali Akbar Roodbari, Ramin Nabizadeh Nodehi, Simin Nasseri, Mohammad Hadil Dehghani, Mahmood Alimohammadi

**Affiliations:** 1 School of Public Health, Tehran University of Medical Sciences, Tehran, Iran; 2 National Institute of Health Research, Tehran University of Medical Sciences, Tehran, Iran; 3 Center for Solid Waste Research, Institute for Environmental Research, Tehran University of Medical Sciences, Tehran, Iran; Plymouth University, United Kingdom

## Abstract

Landfills leachates are known to contain recalcitrant and/or non-biodegradable organic substances and biological processes are not efficient in these cases. A promising alternative to complete oxidation of biorecalcitrant leachate is the use of ultrasonic process as pre-treatment to convert initially biorecalcitrant compounds to more readily biodegradable intermediates. The objectives of this study are to investigate the effect of ultrasonic process on biodegradability improvement. After the optimization by factorial design, the ultrasonic were applied in the treatment of raw leachates using a batch wise mode. For this, different scenarios were tested with regard to power intensities of 70 and 110 W, frequencies of 30, 45 and 60 KHz, reaction times of 30, 60, 90 and 120 minutes and pH of 3, 7 and 10. For determining the effects of catalysts on sonication efficiencies, 5 mg/l of TiO_2_ and ZnO have been also used. Results showed that when applied as relatively brief pre-treatment systems, the sonocatalysis processes induce several modifications of the matrix, which results in significant enhancement of its biodegradability. For this reason, the integrated chemical–biological systems proposed here represent a suitable solution for the treatment of landfill leachate samples.

## Introduction

The generation of leachate remains an inevitable consequence of the practice of waste disposal in sanitary landfills [1]. Leachate from mature landfills contains less biodegradable carbon due to loss from the landfill via methane gas production and is typically characterized by high ammonium (NH_4_^+^) content, low biodegradability (low BOD_5_/COD ratio) and high fraction of refractory and large organic molecules such as humic and fulvic acids [2]. Usually young landfill leachates contain low organic compound concentrations and are treated more easily as compared to the old one [3]. Biodegradable organic compounds and ammonia are leachate constituents that pose the most significant environmental threats [4], [5]. Biological treatment of leachate is often the most cost-effective alternative when compared to other treatment options [6]. Nevertheless, mature leachate effluents are known to contain recalcitrant and/or non-biodegradable organic substances and biological processes are not efficient in these cases [7], [8]. Studies have demonstrated that the major fraction of dissolved organic carbon (DOC) in biologically pre-treated landfill leachates consists of humic substances, mainly in humic and fulvic acids. Traditionally, the degradation of organic compounds and the removal of nitrogen can be achieved by advanced oxidation processes (AOP) [9], [10]. AOP have been used to enhance the biotreatability of wastewaters containing various organic compounds that are non-biodegradable and/or toxic to common microorganisms [11], [12]. Ultrasonic process is one of AOP and involve the generation of the hydroxyl radical (•OH) and pyrolysis phenomenon, which has a very high oxidation potential and is able to oxidize almost all organic pollutants and volatile matter such as NH_3_. Although these processes are very effective in completing mineralization of pollutants, if they are applied as the only treatment process, they will be expensive. A promising alternative to complete oxidation of biorecalcitrant leachate is the use of ultrasonic process as pre-treatment to convert initially biorecalcitrant compounds to more readily biodegradable intermediates, followed by biological oxidation of these intermediates to biomass and water. The major pollutants contained in leachate are biodegradable/non-biodegradable organic material, ammonia and inorganic salts, with anthropogenic organic chemicals, such as phthalates and other endocrine disrupting compounds becoming an increasing concern [13], [14]. Because of the variation in leachate composition and the wide range of pollutants contained in leachate, it is difficult to predict a treatment technique that will be effective for leachate. Usually combinations of physical, chemical and biological methods are used for effective treatment of landfill leachate, since it is difficult to obtain satisfactory results by using any of those methods alone. Sedimentation, air stripping, adsorption, membrane filtration are the major physical methods used for leachate treatment [15], [16]. These methods are usually used in combination with chemical and biological methods. Coagulation–flocculation [17], [18], chemical precipitation [19], [20], chemical–electrochemical oxidations [21], [22] are the major chemical methods used for the landfill leachate treatment. Biological treatment methods used for the leachate treatment can be classified as aerobic, anaerobic and anoxic processes which are widely used for the removal of biodegradable compounds. Physicochemical methods are used along with the biological methods mainly to remove non-biodegradable compounds from the leachate [23], [24], [25]. As a result, parameters have been developed to characterize leachate and predict its treatment efficiency. The ratio of biochemical oxygen demand (BOD) to chemical oxygen demand (COD) (BOD/COD) is a common classification approach. Leachate is classified as stabilized, intermediate, or fresh given BOD/COD values of <0.1, 0.1–0.5, and >0.5, respectively [26], [27], [28]. The BOD/COD ratio indicates that biological processes are appropriate for treatment of fresh leachate because of a higher fraction of biodegradable organic material, while physical–chemical processes are more appropriate for treatment of stabilized leachate because of the high fraction of non-biodegradable organic material. The objectives of this study are to investigate the effect of ultrasonic process on leachate biodegradability improvement.

## Results and Discussion

### Characterization of the Raw Landfill Leachate

Main chemical characteristics of raw leachate summarized in Table 1. With biodegradability ratio (BOD_5_/COD) lower than 0.35 and a pH higher than 8, the samples can be considered as moderately stabilized leachates [29], normally classified as refractory to conventional biodegradation processes. In most cases, intensive and sophisticated physicochemical processes are necessaries for the treatment of aged leachates.

**Table 1:** Chemical characteristics of the studied landfill leachates.

Parameters	Values	Parameters	Values
COD	5691±83	pH	7.9–8.1
Calcium	10.61±0.2	Magnesium	8.65
BOD_5_	1738±36	NH3-N	726±25
TOC	1536±20	TS	1420±29
Alkalinity as CaCO3	3650±123		

Values (except pH) in mg/l.

### Effect of Sonocatalyst on Biodegradability of Leachate

The results indicated that sonocatalyst process can improve leachate biodegradability (BOD_5_/COD ratio). BOD_5_/COD ratio for raw leachate was 0.35 but it reached to 0.786 (with TiO_2_) and 0.783 (with ZnO) after sonication. Independent Samples T-test showed there is significant difference between BOD_5_/COD ratio of raw leachate and pretreated leachate with sonocatalysis process. (p_value_ = 0.000 for both TiO_2_ and ZnO). The results indicated that the system operates with great efficiency (BOD_5_/COD ratio = 0.786) in pH of 10, power of 110 watt, frequency of 60 KHz and TiO_2_ concentration of 5 mg/l.

### Effect of Ultrasound Power Input on Biodegradability Improvement

Figure 1 shows the effect of power input on leachate biodegradability for TiO_2_ and ZnO. As shown in this Figure, the power input clearly improves biodegradability. Independent Samples T-test showed there is significant difference between BOD_5_/COD ratio of raw leachate and pretreated leachate at different powers. (Pvalue = 0.000 for both TiO_2_ and ZnO).

**Figure 1:** BOD/COD ratio input for TiO_2_ and ZnO at different powers (Frequency = 30 KHz, concentration = 5 mg/l, pH = 3).

According to sonochemistry theory, when the ultrasound intensity reaches or exceeds the cavity threshold, bubbles will be formed easily and the cavities collapse violently. Increasing the ultrasonic power will increase the energy of cavitation, lowering the threshold limit of cavitation, and enhancing the quantity of the cavitation bubbles [30]. In other words, at higher intensities, the concentration of hydroxyl radicals and mass transfer are higher which lead to more degradation of organic materials [31] and also more biodegradable intermediate compounds. The efficiency of ratio improvement then increases with the increase of ultrasonic intensity.

### Effect of Exposure Time on Biodegradability Improvement

Results indicated that the exposure time improve biodegradability somehow. Figure 2 shows the effect of exposure time on leachate biodegradability for TiO_2_ and ZnO. As shown in this Figure, the exposure time improve biodegradability somehow. One-Way ANOVA test showed there is no significant difference between BOD_5_/COD ratio of raw leachate and pretreated leachate with sonocatalysis process at different exposure times. (P_value_ = 0.467 for TiO_2_ and 0.398 for ZnO).

**Figure 2:** BOD/COD ratio for TiO_2_ and ZnO at different exposure times (Frequency = 30 KHz, concentration = 5 mg/l, pH = 3).

### Effect of Frequency on Biodegradability Improvement

Figure 3 shows the effect of frequency on leachate biodegradability for TiO_2_ and ZnO. As shown in this Figure, the frequency improves biodegradability. One-Way ANOVA test showed there is significant difference between BOD_5_/COD ratio of raw leachate and pretreated leachate with sonocatalysis process at different frequency. (p_value_ = 0.000 for both TiO_2_ and ZnO). Results of Tukey statistical test also showed that there are significant difference between frequencies of 30 and 60 KHz (P_value_ = 0.000) and 45 and 60 KHz (P_value_ = 0.000).

**Figure 3:** BOD/COD ratio for TiO_2_ and ZnO at different frequencies (power = 70watt, concentration = 5 mg/l, pH = 3).

### Effect of pH on Biodegradability Improvement

Figure 4 shows the effect of pH on leachate biodegradability for TiO_2_ and ZnO. As shown in this Figure, pH improves biodegradability somehow. One-Way ANOVA test showed there is no significant difference between BOD_5_/COD ratio of raw leachate and pretreated leachate with sonocatalysis process at different pH_S_. (p_value_ = 0.503 for TiO_2_ and0.170 for ZnO).

**Figure 4:** BOD/COD ratio for TiO_2_ and ZnO at different pH (power = 70watt, concentration = 5 mg/l, frequency = 30 KHz.

### Effect of Type of Catalysts on Biodegradability Improvement by Ultrasound

Figure 5 shows the effect of types of catalysts on leachate biodegradability (BOD_5_/COD ratio). Results showed that effects of two catalysts on leachate biodegradability was similar but Independent Samples T-test indicated that the there is no significant difference between BOD_5_/COD ratio of raw leachate and pretreated leachate with TiO_2_ and ZnO. (P_value_ = 0.287).

**Figure 5:** BOD_5_/COD ratio for TiO_2_ and ZnO (power = 70watt, concentration = 5 mg/l, frequency = 30 KHz).

### Concurrent Effect of Power Input and Frequency on Biodegradability Improvement by Ultrasound

As mentioned above, power and frequency were effective parameters (statistically significant) on biodegradability improvement by sonocatalysis process. Univeriate statistic test showed that estimates of effect size were 88.6% for power and 74.9% for frequency but concurrent effect was declining (44.4%).

### Biodegradability Changes During Ultrasonic Decomposition

Initially, the biodegradability of the leachates was evaluated through the evolution of the BOD/COD ratio. For untreated samples, this parameter attains values of about 0.35 while ultrasonic treatment of 120 min permit its enhancement up to values near 0.786, which represent substantial biodegradability according to the current literature [32], [33]. This result indicates that the ultrasonic process can break down or rearrange molecular structures of organic matter and convert the non-biodegradable organics to more biodegradable forms. This is a fact of remarkable importance in the case of the application of chemical–biological integrated system to wastewater treatment [33]–[34]. In general, it is admitted that ultrasonic process can transform organic recalcitrant compounds into easily biodegradable products, improving the efficiency and reducing the cost of further biological steps. In a second phase, raw and pre-treated leachate was submitted to a biological degradation process using a sequential batch reactor. The evolution of COD during the biological treatment (figure 6) confirms the low biodegradability of raw leachates, which achieve a maximal COD removal of about 30% at 72 h treatment times. On the other hand, the COD of pre-treated leachates fades progressively attaining COD removal higher than 90% at the end of the 72-h cycle. Additionally, the use of ultrasonically pre-treated samples favored the preservation of physical characteristics of the biological sludge, which could be corroborated by the measurement of traditional physical parameters and microscopic observation [35].

**Figure 6:** Evolution of COD during biological treatment of the leachates (pretreated sample sonicated with power of 110 watt, frequency of 60 KHz, pH of 7 and 5 mg/l of TiO_2_ for 120 minutes).

Landfill leachates contain some macromolecular organic substances that are resistant to biological degradation. With very low biodegradability ratios (BOD/COD), usually lower than 0.35, these complex matrixes show a recognized resistance toward conventional activated sludge systems [36]. When applied as relatively brief pre-treatment systems, the sonocatalysis processes induce several modifications of the matrix, which results in significant enhancement of its biodegradability. For this reason, the integrated chemical–biological systems proposed here represent a suitable solution for the treatment of landfill leachate samples with an efficient remediation of the relevant parameters (COD, TOC).

## Materials and Methods

### Materials

Samples of landfill leachate were obtained from a municipal landfill site (over 10 years old) located in Shahrood (Semnan, Iran). All leachate samples were collected from leachate lift stations or storage tanks, stored at 3°C, and tested within 2 d of collecting the samples. Characteristics of the leachate samples were COD = 5830 mg/l, BOD_5_ = 3940 mg/l, NH_3_-N = 730 mg/l and pH of 8. At the experiments, 5 mg/l of TiO_2_ and ZnO were also been used as catalysts. The ammonia- nitrogen concentrations were analyzed with C_203_ 8 parameter test meter (Hanna electronics co., Ltd.). The pH was measured by a Benchtop pH Meters (Cole-Parmer Co., Ltd).The pH meter was calibrated before each use with pH 3, 7 and 10 buffer solutions. BOD and COD measurements were determined following Standard Methods 5210 and 5220, respectively. Reagents and standard chemicals were purchased from Hach Co., except the BOD buffer solution, which was prepared according to Standard Method 5210. BOD check standards were performed with each batch of BOD measurements [27]. The results were considered good when the value of the BOD check standard fell within the range of 198±30.5 mg/l. The average ± standard deviation of the BOD check standards for the entire duration of the project was 169±29 mg/l, which demonstrates good results given the inherent variability in BOD measurements. COD check standards were also performed with each batch of COD measurements. A COD standard solution of 1000 mg/l was diluted to 200 and 500 mg/l to ensure the accuracy of COD measurements. The relative difference for calibration check standards (RD_cal_) is defined as the absolute difference of the check standard concentration and the known concentration all divided by the known concentration. The RD_cal_ for COD was <10% for the entire duration of the project [28].

### Experimental Set-up

As shown in Figure 7, for the laboratory experiments a cylindrical shape Plexiglas reactor with total volume of 1 L was prepared. The solution in the reactor was mixed with a magnetic stirrer, while sufficient aeration was provided by a compressor connected to a porous stone located in the bottom of the reactor. The compressor was used to ensure completely mixed condition in the reactor. The ultrasonic source was a Model UGMA-5000 ultrasound generator with three 30, 45 and 60 kHz transducers having a titanium probe with 20 mm diameter. The power input could be adjusted continuously from 60 to 120 W. A leachate sample of 1000 ml was sonicated in a covered cylindrical glass vessel. Aeration was supplied by a Model SALWAT air compressor. Samples of activated sludge inoculums were collected directly from the aeration tank of the Shahrood municipal wastewater treatment plant. The sludge was continuously aerated using aeration pumps. Ferrous sulphate (FeSO_4_·7H_2_O), sulphuric acid and hydrogen peroxide (Merck, 30 wt. %) were of analytical grade.

**Figure 7:** Schematic diagram of the reactor.

### Procedure

After the optimization by factorial design, the ultrasonic were applied in the treatment of raw leachates using a batch wise mode. At first, the raw leachate sample was filtered by filter paper (0.45) to remove any suspended solid impurity [28]. Then the sample was adjusted to the required pH with H_2_SO_4_ or NaOH. Then different scenarios were tested with regard to power intensities of 70 and 110 W, frequencies of 30, 45 and 60 KHz, reaction times of 30, 60, 90 and 120 minutes and pH of 3, 7 and 10. For determining the effects of catalysts on sonication efficiencies, 5 mg/l of TiO_2_ and ZnO have been also used. To evaluate the effect of ultrasonic on the biodegradability of raw and sonochemically pre-treated leachates, BOD_5_ and COD of both samples were measured.

### Biological Procedure

The activated sludge system was applied in cylindrical aeration glass-vessels (30 cm of internal diameter and 60 cm of height). The system was aerated by using air pumps placed at the bottom of the reactors. The initial volume of the culture was 150 mL, which was completed to 300 mL with substrates (leachate, pre-treated leachate or glucose) at the beginning of each cycle. The pH was controlled by a probe and adjusted at 7.0 by using H_2_SO_4_ or NaOH. The oxygen concentration was monitored by using an O_2_ probe, located at the top of the reactor. All the experiments were carried out in duplicate and at room temperature (20–25°C) by periods of 72 h. For COD determinations, samples (10 ml each) were taken every 12 h, after they had been centrifuged and filtered through a 0.45 µ Millipore filter [28].

### Ethic Statement

- No specific permits were required for the described field studies.
- No specific permissions were required for these locations/activities.
- Location is not privately-owned or protected in any way.
- The field studies did not involve endangered or protected species.

## References

[1] Hamidi AA, Jyy LT, AbuAhmed MH, Muhammad U, Nordin AM (2011). leachate treatment by swim-bed bio fringe technology.. Desalination.

[2] Anglada Á, Urtiaga A, Ortiz I, Mantzavinos D, Diamadopoulos E (2011). Boron-doped diamond anodic treatment of landfill leachate: Evaluation of operating variables and formation of oxidation by-products. Water Res..

[3] Atmaca E (2009). Treatment of landfill leachate by using electro-Fenton method. J. Hazard. Mater..

[4] Bae BU, Jung S, Kim YR, Shin HS (1999). Treatment of landfill leachate using activated sludge process and electron-beam radiation. Water Res..

[5] Bashir MJK, Hamidi AA, Suffian YM, Qarani AS, Mohajeri S (2010). Stabilized sanitary landfill leachate treatment using anionic resin: treatment optimization by response surface methodology. J. Hazard. Mater..

[6] BenYahmed A, Saidi N, Trabelsi I, Murano F, Dhaifallah T (2009). Microbial characterization during aerobic biological treatment of landfill leachate (Tunisia). Desalination..

[7] Bidhendi ME, Karbassi AR, Baghvand A, Saeedi M, Pejman AH (2010). Potential of natural bed soil in adsorption of heavy metals in industrial waste landfill. Int. J. Environ. Sci. Tech..

[8] Bila DM, Montalvao F, Silva AC, Dezotti M (2005). Ozonation of a landfill leachate: evaluation of toxicity removal and biodegradability improvement. J. Hazard. Mater..

[9] Chen CC (2010). Spatial inequality in municipal solid waste disposal across regions in developing countries. Int. J. Environ. Sci. Tech..

[10] Chianese A, Ranauro R, Verdone N (1999). Treatment of landfill leachate by reverse osmosis. Water Research..

[11] Chiang LC, Chang JE, Wen TC (1995). Indirect oxidation effect in electrochemical oxidation treatment of landfill leachate. Water Res..

[12] Cortez S, Teixeira P, Oliveira R (2011). Manuel Mota, Evaluation of Fenton and ozone-based advanced oxidation processes as mature landfill leachate pre-treatments. J. Environ. Manage..

[13] deMorais JL, Zamora PP (2005). Use of advanced oxidation processes to improve the biodegradability of mature landfill leachates. J. Hazard. Mater..

[14] Guo JS, Abbas AA, Chen YP, Liu ZP, Fang F (2010). Treatment of landfill leachate using a combined stripping, Fenton, SBR, and coagulation process. J. Hazard. Mater..

[15] Kargi F, Pamukoglu MY (2003). Removal of Cu(II) ions by biosorption onto powdered waste sludge (PWS) prior to biological treatment in an activated sludge unit: A statistical design approach. Process Biochem..

[16] Kargi F, Pamukoglu MY (2004). Repeated fed-batch biological treatment of pre-treated landfill leachate by powdered activated carbon addition. Enzyme Microb. Technol..

[17] Kurniawan TA, Lo WH (2009). Removal of refractory compounds from stabilized landfill leachate using an integrated H_2_O_2_ oxidation and granular activated carbon (GAC) adsorption treatment. Water Res..

[18] Leao S, Bishop I, Evans D (2004). Spatial-Temporal model for demand and allocation of waste landfills in growing urban region. Computers, Environ. Urban Sys..

[19] Li HJ, Gu YY, Zhao YC, Wen ZP (2010). Leachate treatment using a demonstration aged refuse biofilter. J. Environ. Sci..

[20] Lim PE, Lim SP, Seng CE, Noor MdA (2010). Treatment of landfill leachate in sequencing batch reactor supplemented with activated rice husk as adsorbent. Chem. Eng. J..

[21] Lim YN, Shaaban MdG, Yin CY (2009). Treatment of landfill leachate using palm shell-activated carbon column: Axial dispersion modeling and treatment profile. Chem. Eng. J..

[22] Mahini AS, Gholamalifard M (2006). Siting MSW landfills with a weighted linear combination methodology in a GIS environment. Int. J. Environ. Sci. Tech..

[23] Ogundiran OO, Afolabi TA (2008). Assessment of the physicochemical parameters and heavy metals toxicity of leachates from municipal solid waste open dumpsite. Int. J. Environ. Sci. Tech..

[24] Pattnaik S, Reddy MV (2010). Assessment of municipal solid waste management in Puducherry (Pondicherry) India. Resour. Conserv. Recycl..

[25] Pilli S, Bhunia P, Yan S, LeBlanc RJ, Tyagi RD (2011). Ultrasonic pretreatment of sludge: A review. Ultrason. Sonochem..

[26] Pi KW, Li Z, Wan DJ, Gao LX (2009). Pretreatment of municipal landfill leachate by a combined process. Process Saf Environ..

[27] Robinson HD, Maris PJ (1983). Treatment of leachates from domestic wastes in landfills–I: Aerobic biological treatment of a medium-strength leachate. Water Res..

[28] Schoeman JJ (2008). Evaluation of electrodialysis for the treamnet of a hazardous leachate. Desalination..

[29] Schuk WW, James SC (1986). Treatment of landfill leachate at publicly owned treatment works. Wast. Manag. Res..

[30] Scullion J, Winson M, Matthews R (2007). Inhibition and recovery in a fixed microbial film leachate treatment system subject to shock loading of copper and zinc. Water Res..

[31] Sun YJ, Ma GP, Ye XQ, Kakuda Yk, Meng RF (2010). Stability of all-trans-β-carotene under ultrasound treatment in a model system: Effects of different factors, kinetics and newly formed compounds. Ultrason. Sonochem..

[32] Suthar S, Singh S (2008). Vermicomposting of domestic waste by using two epigeic earthworms (Perionyx excavatus and Perionyx sansibaricus). Int. J. Environ. Sci. Tech..

[33] Vilar VJP, Rocha EMR, Mota FS, Fonseca A, Saraiva I (2010). Treatment of a sanitary landfill leachate using combined solar photo-Fenton and biological immobilized biomass reactor at a pilot scale. Water Res..

[34] Dehghani MH, Mahvi AH, Jahed GR, Sheikhi R (2007). Investigation and evaluation of ultrasound reactor for reduction of fungi from sewage. JZUSB.. 8(7) 493–498.

[35] Mahvi AH (2009). Application of ultrasonic technology for water and wastewater treatment. IJPH.. 38(2) 1–9.

[36] Mahvi AH, Maleki A, Rezaee R, Safari M (2009). Reduction of humic substances in water by application of ultrasound waves and ultraviolet irradiation. IJEHSE.. 6(4) 233–238.

